This article has been retracted.

# Detection and Prediction of Peripheral Arterial Plaque Using Vessel Wall MR in Patients with Diabetes

**DOI:** 10.1155/2021/5585846

**Published:** 2021-04-24

**Authors:** Li Wang, Wei Deng, Jianke Liang, Weizhao Zhuang, Huigang Feng, Gaoming Zhuang, Dexiang Liu, Hanwei Chen

**Affiliations:** ^1^Department of Radiology, The First Affiliated Hospital, Jinan University, Guangzhou, China; ^2^Department of Radiology, Guangzhou Panyu Central Hospital, Guangzhou, China; ^3^Medical Imaging Institute of Panyu, Guangzhou, China; ^4^Invasive Technology Department, Guangzhou Panyu Central Hospital, Guangzhou, China; ^5^Invasive Technology Department, The First Affiliated Hospital, Jinan University, Guangzhou, China

## Abstract

**Objectives:**

To evaluate the predictive performance of a newly developed delay alternating with nutation for tailored excitation (DANTE) pulse sequence for detecting lower extremity artery wall morphology and distribution in patients with peripheral artery disease (PAD) with diabetes.

**Methods:**

Seventy-four PAD patients diagnosed according to 2011 WHO criteria were enrolled, who has diabetic diagnosis by 1999 WHO diabetes criteria. All patients received sequential DANTE, T2WI, DANTE-enhance, and CE-MRA scans. The images consisted of three parts: the iliac artery (segment 1), femoral artery (segment 2), and popliteal artery (segment 3). Regions of interest (ROIs) were drawn on vessels, muscle, and background, and multiple imaging metrics compared between modalities, including image quality score, image noise, signal-to-noise ratio (SNR), and contrast-to-noise ratio (CNR). In the images with a score greater than 2, the lumen area (LA), total vessel area (TVA), and vessel thickness (VT) can be identified using semiautomatic image analysis vessel morphology parameters.

**Results:**

All 222 arterial segments were successfully analyzed from 71 patients, after exclusion of three subjects with poor image quality (IQ < 2) in segment 3. There were 54 diabetic and 17 nondiabetic patients. Quantitative analysis shows that the CNR difference between diabetic patients and nondiabetic patients was statistically significant for the same segment, while there was no significant difference among the three segments of SNR and CNR. There were a total of 54 diabetics with plaque distribution data, which showed that LA of segments 1 and 2 was higher than that of segment 3. The VWI of segments 1 and 2 was lower than segment 3. Diabetic was associated with vascular WT 3 and WA3, which increased by 0.23 and 0.83 units on average compared without diabetic foot, respectively. Diabetic foot was associated with vascular WT 3, which increased by 0.37 units on average compared without diabetic foot. The incidence of segment 3 plaques was higher than that of segment 1. The incidence of the left and right plaques was different.

**Conclusions:**

MR imaging using the DANTE and multicontrast sequence could evaluate plaque morphology, and distribution of lower extremities and the occurrence of diabetic foot development are closely related; it may predict occurrence of PAD with diabetic foot.

## 1. Introduction

Approximately 120 million people in China are currently affected by patients with diabetes, which has resulted in an 11.6% incidence in China. The number of people with the disease is the highest in the world [1]. The incidence of peripheral artery disease (PAD) in diabetic patients is twice as high as in nondiabetic patients [2]. The prevalence rate of PAD in type 2 diabetes patients over 50 years old was 21.2% [3]; PAD of lower extremity arterial lesions is one of the most important pathogenesis of diabetic foot. PAD was present in 47.5% of diabetic foot patients among patients with diabetes. The results of two surveys on diabetic foot in China in 2004 and 2012 showed that the combined PAD of diabetic foot was 62.9% and 59%, respectively, indicating that the combined PAD of diabetic foot is one of the important causes of diabetic foot ulcer (DFU) [4]. Diabetic foot is one of the main causes of disability and death in diabetic patients. At the same time, the symptoms of PAD with diabetes are more insidious and atypical because of its pathological and anatomical characteristics and various pathogenic factors. At present, the rate of PAD diagnosis and treatment of diabetes is low, which is often ignored by the clinic. The rate of missed diagnosis reaches 55.7%, leading to a high incidence of foot ulcer, amputation rate, and mortality of diabetic patients. PAD China's prevention and cure of diabetic foot patients with diabetes guide (2019 edition) (II) [5, 6] points out that early diagnosis and intervention of the PAD are the key to the prevention of diabetic foot, and its prognosis predictions may have some significance.

Cardiovascular magnetic resonance imaging (MRI), particularly high-resolution black-blood MRI, is a promising noninvasive modality for evaluating vessel arterial wall imaging (VWI) and plaque morphology owing to its high spatial resolution, flexibility, and safety, which completely suppresses blood flow signals in the blood vessel cavity and soft tissue signals around the blood vessels to show the vessel wall thickness and plaques burden. In particular, dark-blood MRI is widely used to measure plaque volume and composition (fibrous cap, lipid-rich core, intraplaque hemorrhage, and calcification) during cardiovascular disease progression [7–10]. MRI VWI can not only identify arterial vascular plaques throughout the body but also accurate identification of unstable plaque morphology.

High-resolution MR wall imaging adopts blood flow inhibition technology, which can accurately and intuitively show the morphology of arterial wall and plaque signs and plaque components. Spatial saturation pulse, also known as saturation band method [11], is widely used in clinical practice due to its simple operation and short suppression time of blood flow. However, it is hard to completely suppress the abnormal slow flow of blood signal caused by eddy or turbulence. Double inversion recovery (DIR) is considered the standard method of MRI black-blood technique, but the blood flow signal with slow or turbulent flow cannot be completely suppressed. Four reinversion recoveries (QIR) are mainly used to enhance the imaging of the vessel wall and cannot completely suppress the signal of slow blood flow. Variable inversion three-dimensional fast spin echo technology (SPACE) with angle and long echo chain. This imaging method has a high resolution and can be reassembled in any plane. However, its gradient magnetic field is insufficient to suppress complex blood flow signals [12, 13]. Motion-sensitive driven balance (MSDE) sequence can inhibit slow blood flow, but T2 signal attenuation leads to signal loss [14]. Improved motion-sensitive driven balance (iMSDE) sequence can improve image signal-to-noise ratio (SNR), which reduces the impact caused by slow blood flow, but the left signal loss is still less [15].

Li et al. [16] reported that delayed alternating nutation adjustment excitation (DANTE) in 2012, the method is a nonselective unbalanced RF pulse balanced steady-free precession sequence. With nonselective RF pulses, longitudinal magnetization of static tissues is retained to the maximum extent, which can attenuate the blood flow largely or completely. DANTE inhibits slow blood flow in all directions (>0.1 cm/s), which can be used for 3D acquisition. The sequence is less sensitive to magnetic field heterogeneity and lower damage of signal. It is proposed that the DANTE sequence could be applied to black-blood vessel imaging of the carotid artery wall [17], and a recent study demonstrated the applicability of the DANTE sequence for identification of atherosclerotic plaques with PAD [18].

The aim of this study was to assess the diagnostic performance of DANTE sequence for detecting PAD in patients with diabetes in early and to assess the prognosis of diabetic foot.

## 2. Materials and Methods

### 2.1. Patients

This study was approved by the hospital's review board. Informed consent was obtained from all patients. From May 2018 through October 2020, 71 subjects were identified from consecutive patients with according to criteria [19] and who have diabetes diagnosis by 1999 WHO diabetes criteria [20]. All patients exhibited intermittent claudication with/without critical limb ischemia.

### 2.2. MRI

The MRI examinations were performed using a 1.5 T scanner (MAGNETOM Avanto, Siemens Healthcare, Erlangen, Germany). Patients were placed in the supine position and bilateral legs imaged foot-first using sixteen element peripheral vascular coils. Scans were conducted in three segments. Multicontrast sequence was performed by the same coils used in both scans.

### 2.3. DANTE

The 3D imaging volume was prescribed to cover the calves on a scout scan. A true FISP sequence was performed first, followed by 2D-TSE T2-weighted (T2WI) axial scanning. The parameters for DANTE were as follows: flip angle = 15°, pulse train length = 125, voxel size = 0.7 × 0.7 × 0.7 mm^3^, TR/TE = 600/18 ms, and acceleration factor = 60.

### 2.4. CE-MRA

Contrast-enhanced MRA was performed after DANTE MRI. The scanning range and coils were the same as for DANTE MRI. During intravenous administration of gadopentetate dimeglumine (Gd-DTPA, MagnevistVR, Schering AG, Berlin, Germany), collecting the coronal image. Relevant imaging parameters of DANTE were as follows: TR/TE = 600/18 ms, flip angle = 25°, and voxel size = 0.7 × 0.7 × 0.7 mm^3^. Using a time-resolved axial scan confirm the contrast transit time from the radial vein to the common femoral arteries following the administration of a 2 mL test bolus. Gd-DTPA was administered at a dose of 0.2 mmol/kg bodyweight using an automated injector (Magenvist, Bayer Schering, Berlin, Germany). The injection rate (2 to 2.5 mL/s) was modified to cover 70% of the total acquisition time and following about 20 mL saline flush the tubing at the same rate for the 30% remaining time period. Scanning time was 5 m 18 s for each segment, and scanning scope was 50 cm per segment.

### 2.5. Image Analysis

Images were transferred to a workstation (Siemens, Germany); Carestream Vue PACS and multiplanar reformation (MPR) were used to match cross-sectional images for postprocessing. Two radiologists (L.W. and W.D) with 10 and 17 years' experience, respectively, in cardiovascular MR imaging evaluated the images. The lower extremity artery network was divided into three parts, including segments of the iliac artery (segment 1: bilateral common ilium artery, the internal ilium artery, and the external ilium artery), femoral artery (segment 2: bilateral common femoral artery, the superficial femoral artery, and deep femoral artery segment), and popliteal artery (segment 3: bilateral popliteal artery, tibialis anterior and posterior arteries, and fibularis artery).

We evaluated image signal-to-noise ratio (SNR), which measured arterial signal intensity divided by the calculated noise define as a quantitative evaluation. Artery tissue contrast-to noise ratio (CNR), which measured the difference in signal intensity between arterial signal intensity and the surrounding muscle tissue divided by the calculated noise.

Image quality (IQ) was assessed using a previously developed four-point scale (1 = unidentifiable arterial wall and lumen margins; 2 = visible arterial wall with obscured substructures; 3 = minimal motion or flow artifacts, identifiable vessel wall, and lumen boundaries; and 4 = no artifacts, detailed description of wall architecture, and plaque composition) [21] (Figure 1). Poor image quality was excluded which unidentified lumen and vessel wall. In the images with quality scores greater than 2, the lumen area (LA), total vessel area (TVA), vessel thickness (VT) can be identified using semiautomatic image analysis software Carestream Vue PACS. We derived the wall area (WA = VA − LA) and mean/maximum wall thickness (MeanWT, MaxWT, and MinWT) from the LA. The MeanWT for each location was calculated by (MaxWT − MinWT)/MaxWT, VWI = WA/TVA. The region of interest (ROI) was drawn three times at different sites and the average calculated for each parameter.

Outline intraplaque hemorrhage (IPH), lipid-rich necrotic core (LRNC), and calcification (CA) were based on previously published carotid CMR criteria for imaging with multicontrast techniques [22] (Table 1**).**

To discuss the effect of patient characteristics on the image quality of DANTE, we performed a subgroup analysis above in patients with and without diabetic foot.

### 2.6. Statistical Analysis

Data analysis was performed using SPSS for R version 3.6.3. The analysis was oriented for a normality test statistically (Shapiro-Wilk test). Among 71 subjects, to compare the quantitative measurements, SNR and CNR from diabetic and nondiabetic patients, Mann-Whiney *U*-test was performed for evaluating the difference in each arterial segments. For the comparison of SNR and CNR among the three segments and LV, WA, WT, and VWI of a diabetic, a nonparametric test (Kruskal-Wallis *H*-test) was used to assess differences. The characteristics of plaque distribution in diabetic patients were assessed with the Fisher test. Correlation analysis between diabetic, diabetic foot, and WT, WA, and VWI was performed. The *p* value < 0.05 was considered a significant difference.

## 3. Results

All 222 arterial segments were successfully analyzed from 71 patients, after exclusion of three subjects with poor image quality (IQ < 2) in segment 3. The study population is presented by demographic data in Table 2. There were 54 diabetic and 17 nondiabetic patients. As can be seen from the MRI images in Figures 2–4, the arterial vessel walls of the lower extremities of different type 2 diabetic patients could be clearly visualized using the DANTE sequence.

Further, we analyzed the data related to MRI images. To compare the differences of SNR and CNR in the same segment between diabetic and nondiabetic patients, Mann-Whiney *U*-test was performed. Quantitative analysis showed that the CNR difference between diabetic patients and nondiabetic patients was statistically significant for the same segment (−4.90 ± 6.56 vs. −1.13 ± 5.31; *p* < 0.006), and it could be considered that the CNR of diabetic patients was lower than that of nondiabetic patients in Figure 5.

Kruskal-Wallis *H*-test was performed on SNR and CNR of the three segments with diabetes to compare the differences of SNR and CNR of the three segments. There was not statistically significant, so the three segments of SNR and CNR could not be considered to be different (*p* > 0.05) (Table 3).

Correlation analysis was performed between whether a person has diabetes/diabetic feet and plaque and component plaque (Figure 6). Firstly, the WT, WA, and VWI are analyzed. There were a total of 54 diabetics with plaque distribution data, comparison of plaque morphology, and components in different arterial segments. Tukey's test showed that the LA of segments 1 and 3 and segments 2 and 3 were statistically significant (*p* < 0.001, *p* = 0.02), respectively. The LA of segment 1 was higher than that of segment 3, and the LA of segment 2 was higher than that of segment 3. Tukey's test showed that the VWI of segments 1 and 3 and segment 2 and 3 was statistically significant (*p* = 0.0021, *p* = 0.03), respectively. The VWI of segment 1 was lower than segment 3, and the VWI of segment 2 was lower than segment 3. Then, the VT, WA, and VWI were taken as dependent variables and diabetes/diabetic foot as independent variables, linear regression was performed. Diabetes was associated with vascular VT 3 and WA3, which increased by 0.23 and 0.83 units on average compared without diabetic foot, respectively (*p* = 0.04, *p* = 0.01) (Table 4).

Diabetic foot was associated with vascular WT 3, which increased by 0.37 units on average compared without diabetic foot (*p* = 0.046).

Fisher's test was used to compare the plaque incidence of the three segments in pairs. Bonferroni's method was used to correct the test level (0.05/3 = 0.017). It was statistically significant that the incidence of segment 3 plaques was higher than that of segment 1 (*p* < 0.017) (Table 5). The incidence of plaque at different segments was tested using Fisher's test. It could not be considered that the incidence of the left and right plaques was different (*p* = 0.23). The kappa value for interobserver agreement between the two readers was 0.95.

## 4. Discussion

We evaluated the diagnostic performance of the newly developed DANTE black-blood MRI technique for the large coverage detection of whole lower peripheral in patients with diabetes. Accurate evaluating is essential, as prognosis and management of patients with diabetic is related to the plaque morphology and distribution. Multicontrast MR vessel wall imaging techniques, which include morphological DANTE imaging, T2WI, DANTE-enhance, and CE-MRA, have been proven to improve accuracy therapy of early-stage diabetes and have shown potential in monitoring treatment response to prevent diabetic foot.

Black-blood MRI is widely applied for intracranial imaging to noninvasively evaluate plaque morphology, composition, and stability [23]. However, due to the lower peripheral blood flow, with the advent of black-blood MRI imaging, it is impossible to image the whole lower peripheral arteries except for the femoral artery [24]. DANTE translates to a consistently good quality of flow signal suppression even if the blood flow is rather slow in the stenotic peripheral arteries. Both arterial and venous blood flows are completely suppressed. More importantly, DANTE is insensitive to B1 field inhomogeneity and independent of the inflow effect. In this study, isotropic spatial resolution and about 90 cm longitudinal coverage (each segment is 352 mm, 3 segments, overlapping 10%) is feasible in a short time of less than 6 min; we acquired excellent imaging with high SNR and CNR. The shorter coverage, in contrast, would demand over 20 minutes for the commonly used method 2D sequence [18]. Comparable with other 3D sequence, studies show excellent results [25–27]. The DANTE using lower refocusing flip-angles could enhance this effect and long echo trains that induce larger phase dispersion. We acknowledge that in-flow of inverted blood spins would not be sufficient with this thickness and would give way quality of black-blood efficiency for the slices at flow downstream. In our study, we measure vessel wall with resolution of 0.7 × 0.7 × 0.7 mm^3^, better than resolution of 0.78 × 0.49 × 2 mm^3^ with MRI and 3D TOF [28]. Further, images acquired using DANTE were of comparable quality to T2WI and demonstrated sufficient signal suppression for thin layer scanning. These features gave rise to high diagnostic performance of DANTE.

We evaluate the different segments of imaging quality in diabetic and nondiabetic patients; the slightly lower image quality show that the second segment SNR of the diabetic group was lower than that of non-diabetic foot; CNR in the third segment was lower than that in the nondiabetic group; and comparison of SNR and CNR of different arterial segments in diabetic was done. In addition, we assessed three segments by comparing their LA, WA, WT, and VWI in patients with diabetes, and different segments had a significant effect on LA, because LA may taper from proximal to distal. In this study, LA of the 3rd segment is smallest. There are significant effects VT-3 and WA-3 in diabetic foot compared with that in nondiabetic foot, respectively. VT of diabetic foot was higher than without the diabetic foot. Foot artery of diabetic foot was smaller vessel area than nondiabetic foot; the result was similar with previous study [29]. Plaque morphology and distribution of lower extremities and occurrence of diabetic foot development are closely related. These results suggest that lower extremity arterial stenosis and diabetic foot. The result was mainly caused by diabetes with atherosclerotic risk factors.

There were several limitations to this study. First, the sample size was small and the cross-section observational design did not allow for assessment of PAD with diabetic progression. Larger scale studies including healthy controls are required for comparison and assessment of reproducibility. Second, plaque structure and composition were unclear below the popliteal artery, so improved image SNR is still required for assessment of small arterial branches. Third, only the effect of diabetic foot on image quality was analyzed.

Further studies should be performed to investigate the relationship between image quality and other patient characteristics such as age, blood sugar level, hypertension, and heart attack.

## 5. Conclusions

Magnetic resonance imaging using the DANTE sequence is a feasible modality for quantitative analysis of lower extremity vessel wall morphology and detection of plaque components, with accuracy comparable to T2WI. Larger scale studies are warranted to confirm the diagnostic accuracy for atherosclerotic plaques in clinical practice.

## Figures and Tables

**Figure 1:** Measured lumen and vessel wall.

**Figure 2:** Magnetic resonance images of the lower extremity arteries of a 84-year-old male patient with calf arterial disease and type 2 diabetes using of DANTE sequence. Both cross-sectional images clearly reveal the vessel wall (yellow arrows). (a) MRA. (b) DANTE. (c) 2D-TSE. (1) The right superficial femoral artery. (2) Popliteal artery. (3) Left PTA.

**Figure 3:** Magnetic resonance images of the lower extremity arteries of a 42-year-old male patient with calf arterial disease and hypertension using of DANTE sequence. Both cross-sectional images clearly reveal the left iliac external artery vessel wall. (a) DANTE. (b). 2D-TSE.

**Figure 4:** Lower extremity vascular images of a 69-year-old male with calf arterial disease and type 2 diabetes. Representative plaque from the left superficial femoral artery (red arrows). (a) Image using DANTE. (b) CE-MRA image.

**Figure 5:** Comparison of SNR (a) and CNR (b) of arterial segments in 71 patients with diabetes and without diabetes. ^∗∗^*p* < 0.01 vs. the nondiabetic group. SNR: signal-to-noise; CNR: contrast-to-noise ratio.

**Figure 6:** Comparison of plaque morphology and components in different arterial segments with diabetic. ^∗^*p* < 0.05 and ^∗∗^*p* < 0.01 vs. the segment 1 group. ^#^*p* < 0.05 vs. the segment 2 group.

**Table 1:** MRI signal features noted for the identification of atherosclerotic plaque constituents.

Multicontrast sequences				
Plaque composition	TOF	T1	PD	T2
Calcification	−	−	−	−/+
Lipid core	O	+	+	−/o
Hemorrhage	−	−		−
Acute (<1 week)	+	+	O	O
Recent (1-6 weeks)	+	+	+	+
Fibrous constituent	O/+	O/+	O/+	O/+

Compare the muscle: +: Hpersignal; O: Isosignal; −: Hpeosignal.

**Table 2:** Demographic data in study population with and without diabetes.

Characteristics	Patients with diabetes (*n* = 54)	Patients without diabetes (*n* = 17)	*p* value
Age (years)	51.69 ± 19.96	68.81 ± 11.46	0.033
Sex (male/female)	37/20	11/6	0.757
Systolic blood pressure (mmHg)	137 ± 30/80 to 180	125 ± 18/110 to 140	0.019
Diastolic blood pressure (mmHg) intermittent claudication	81 ± 12/66 to 98	88 ± 11/75 to 96	0.021
Rest pain	25 (44%)	8 (47%)	0.087
Diabetic foot	20 (35%)	9 (53%)	0.096
Amputation (unilateral leg)	2 (4%)	0	0.363
Vascular malformation	0	3 (18%)	0.355
Smoking	16 (28%)	5 (29%)	0.546
Coronary heart disease (CHD)	15 (26%)	8 (47%)	0.225

Values are mean ± SD or *n* (%).

**Table 3:** Comparison of SNR and CNR of different arterial segments in diabetic.

Variate	Segment 1	Segment 2	Segment 3	*p* value
	(*n* = 54)	(*n* = 54)	(*n* = 54)	
SNR	55.65 ± 14.58	56.77 ± 21.45	67.06 ± 14.09	0.12
CNR	−8.66 ± 8.38	−5.66 ± 7.68	−5.01 ± 7.26	0.42

Values are mean ± SD.

**Table 4:** Correlation of plaque morphology and components with diabetic/diabetic foot.

Variate	Nondiabetic	Diabetic	Effect value	*p* value	Nondiabetic foot	Diabetic foot	Effect value	*p* value
	(*n* = 17)	(*n* = 54)			(*n* = 50)	(*n* = 21)		
VT-1	0.95 ± 0.55	1.09 ± 0.57	0.04	0.83	0.96 ± 0.53	1.17 ± 0.75	0.04	0.89
VT-2	1.87 ± 4.54	1.17 ± 0.64	-1.41	0.37	1.71 ± 4.22	1.77 ± 1.20	-0.61	0.75
VT-3	1.11 ± 0.51	1.45 ± 0.55	0.23	0.04	1.12 ± 0.51	1.74 ± 0.37	0.37	0.046
WA-1	20.31 ± 12.24	23.40 ± 15.04	3.98	0.37	20.23 ± 12.33	27.50 ± 16.37	5.67	0.30
WA-2	16.53 ± 9.72	16.07 ± 5.77	-2.72	0.42	15.56 ± 7.10	23.56 ± 17.29	5.75	0.16
WA-3	13.74 ± 6.89	17.22 ± 7.30	0.83	0.01	13.91 ± 6.72	19.78 ± 8.34	2.73	0.32
VWI-1	0.37 ± 0.18	0.41 ± 0.23	0.05	0.50	0.38 ± 0.19	0.42 ± 0.23	0.01	0.87
VWI-2	0.52 ± 0.16	0.53 ± 0.15	-0.04	0.48	0.51 ± 0.15	0.61 ± 0.21	0.04	0.56
VWI-3	0.56 ± 0.19	0.71 ± 0.16	0.09	0.13	0.57 ± 0.19	0.78 ± 0.11	0.11	0.11

**Table 5:** Comparison with incidence of plaque at different segments.

Segment	Segment 1	Segment 2
Segment 2	0.56	—
Segment 3	0.009	>0.99

## Data Availability

The data that support the findings of this study are available on request from the corresponding author. The data are not publicly available due to records which may contain information that could compromise patient confidentiality.
